The article "Method for Forecasting Urban National Sports and Fitness Demand Based on Ant Colony Algorithm" was published in 2021. Journal: Comput Intell Neurosci.

# Method for Forecasting Urban National Sports and Fitness Demand Based on Ant Colony Algorithm

**DOI:** 10.1155/2021/5917756

**Published:** 2021-12-24

**Authors:** Jianhui Wu

**Affiliations:** Department of Physical Education, Gannan Normal University, Ganzhou 341000, China

## Abstract

With the continuous development of social economy, when people are pursuing economic income, they are also gradually paying attention to their own physical health. They achieve their own physical exercise through sports such as running, fitness, and mountaineering, but these sports often require a certain venue and equipment. Therefore, in view of these sports fitness demands, the ant colony algorithm is introduced to sort out the fitness activities in the context of urban residents' supply and demand relationships, analyze the demand from both subjective and objective aspects, and explore the lack of supply of sports facilities in this paper. Analysis is conducted from cognitive and national fitness, social needs, habits, and other perspectives. It tries to guide the rational allocation and creation of resources, obtain residents' fitness awareness and support, and provide corresponding suggestions and support for residents' fitness activities. The simulation experimental results show that the ant colony algorithm is effective and can support the predictive analysis of the urban national fitness demand.

## 1. Introduction

With the continuous development of social economy, people also attach great importance to physical health, especially for urban residents in agglomerations, and their demand for urban sports venues and sports facilities is also increasing [1–3]. The construction of sports facilities is directly related to the way of urban residents' physical exercise and related enthusiasm [4, 5]. For urban residents, the development of natural resources of land and the construction of urbanization have significantly increased the scope and degree of development of the city. In addition, due to the influence of traditional concepts, there is no probability of dedicated land for sports facilities; especially, the increase in population size has further compressed the living space. [6, 7] However, in recent years, with the inclination and implementation of policies such as sports power, urban residents' exercise methods have changed in many ways, such as indoor yoga, rock climbing, fitness, outdoor mountaineering, and marathons, which have gradually become the interaction between people and space, and more urban residents have corresponding choices from indoor to outdoor environments [8, 9].

Under the conditions of haze, strong wind, heavy rain, snow, etc., it is a challenge for outdoor sports. Therefore, indoor fitness has become an alternative to sports fitness. Because it is not affected by the external environment but only subjects to the choice of the indoor environment. This method allows residents not only to perform corresponding physical fitness exercises but also to have social skills and methods [10, 11]. In view of these needs and limitations, the ant colony algorithm is introduced in this paper to sort out the physical fitness needs of urban residents in the supply and demand relationship, analyze the demand from both subjective and objective perspectives, try to explore the allocation of corresponding fitness resources, and respect the opinions of the corresponding urban residents, to provide support and suggestions for urban residents' physical fitness, aiming to improve the popularity and effectiveness of sports for all.

## 2. Ant Colony Algorithm

For the ant colony algorithm, it has distributed and heuristic-related characteristics, which is an algorithm of continuous learning, continuous iteration, and continuous enhancement. The execution process of the ant colony algorithm mainly has two steps of adaptation and cooperation [12, 13].

The ant colony algorithm was originally a solution model proposed for the TSP problem. Its main purpose is to solve the Hamiltonian circuit in the entire graph. It traverses all the nodes and solves the shortest length.

At the beginning of the initialization, the ants start to select the corresponding starting point and then enter the adaptation phase, that is, to find the corresponding path, they are proceeded according to the following rules:

For ant *k*, the probability of selecting city *j* from city *i* at time *t* is expressed by the following formula:

(1) $$\begin{array}{c} p_{ij}^{k}\left(t\right)=\left\{\begin{array}{c} \frac{{\left[\tau_{ij}\left(t\right)\right]}^{\alpha }\cdot {\left[\eta_{ij}\left(t\right)\right]}^{\beta }}{\sum_{k\in {\text{allowed}}_{k}}{\left[\tau_{ij}\left(t\right)\right]}^{\alpha }\cdot {\left[\eta_{ij}\left(t\right)\right]}^{\beta }},\;j\in {\text{allowed}}_{k},\\ 0,\;\text{otherwise.} \end{array}\right. \end{array}$$

In the above formula, *τ*_*ij*_(*t*) represents the concentration of pheromone on the edge (*i*, *j*) at time *t*, *η*_*ij*_=1/*d*_*ij*_ is used to represent the heuristic factor. The larger *d*_*ij*_, the smaller heuristic factor, and the smaller probability of the ant choosing this path among many paths.*α* represents the heuristic factor of the pheromone, which is the effect of the information generated by the ant during the entire search process. If the value of *α* is larger, it indicates that the ant is more inclined to choose the path searched by other ants. All ants will search and traverse all nodes according to formula (1), and there will be *m* circuit solutions for *m* ants [14, 15].

The collaboration stage points mainly that ants treat the pheromone left by themselves in the search process as the basis for next round of ant searching iterative solution. The pheromone solution rule formula is as follows:

(2) $$\begin{array}{c} \tau_{ij}\left(t+1\right)=\left(1-\rho \right)\cdot \tau_{ij}\left(t\right)+\sum_{k=1}^{m}\Delta \tau_{ij}^{k}. \end{array}$$

Among them, *ρ* represents the pheromone volatilization factor, and Δ*τ*_*ij*_^*k*^ represents the pheromone released by ant *k* at edge (*i*, *j*) the last time, as shown in the following formula:

(3) $$\begin{array}{c} \Delta \tau_{ij}^{k}=\left[\begin{array}{c} \frac{1}{C^{k}},\;\left(i,j\right)\in T^{k},\\ 0,\;\text{otherwise.} \end{array}\right] \end{array}$$

Among them, *C*^*k*^ represents the overall length of the path *T*^*k*^ that the ant *k* is looking for from *t* to *t* + 1. It can be seen from formula (3) that the smaller the *C*^*k*^ value, the larger the increment of pheromone on the path *T*^*k*^, and larger the probability of the path being selected by next iteration [16, 17].

There are certain shortcomings for the ant colony algorithm in processing large-scale spatial data: (1) the path chosen by all ants will be affected by the size of the pheromone produced in the previous iteration, so in the continuous search process, a local optimum is easily produced; (2) during the execution of the ant colony algorithm, the path chosen by the ants is random, and it is relatively difficult to choose a shorter path among many paths, so the algorithm execution process is more time consuming.

The problem of facility location has been around for a long time. As a basic facility location model, the P-median location problem has been applied to many occasions. The P-median location problem is to find *p* median locations from *N* sets as various types. The median of the set of median points is *M*, and all demand points are allocated to only one class so that the sum of the distances from each demand point to the median point in the class is minimized. The P-median problem is also called the minimum sum problem.

The neutral problem can be expressed by the following mathematical formulas, specifically as shown in the following formulas:

(4) $$\begin{array}{c} Z_{\min}=\sum_{i\in M}\sum_{j\in N}d_{ij}x_{ij}, \end{array}$$

(5) $$\begin{array}{c} \sum_{i\in N}x_{ij}=1,\;i\in N, \end{array}$$

(6) $$\begin{array}{c} x_{ij}=0,\;k\in N-M, \end{array}$$

(7) $$\begin{array}{c} \sum_{j\in M}x_{jj}=p,\;j\in M, \end{array}$$

(8) $$\begin{array}{c} x_{ij}\in \left\{0,1\right\},\;i\in N,j\in M. \end{array}$$

In the above formula, *Z* represents the objective function value, *d*_*ij*_ represents the distance from *i* in the set *N* to *j* in the neutral set *M*, and *x*_*ij*_ indicates whether *i* belongs to *j*. If it belongs to j, it is 1; otherwise, it is 0.

In recent years, the P-neutral problem is still a research hotspot. At the same time, many variants of the P-neutral problem have appeared, such as the dynamic P-neutral problem [18, 19].

Firstly, the corresponding investigations, statistical analysis, and other methods are adopted for research, relying on the ant colony algorithm and comprehensively integrating quantitative and qualitative methods. Secondly, the final result is obtained from the investigation and research, and communication of the corresponding community residents, as shown in Figure 1.

### 2.1. Expert Consultation

According to relevant research, experts and scholars in sports, medical care, planning, community workers, urban management, etc., are selected to conduct comprehensive interviews to fully understand the issues and factors that urban residents need to consider in physical fitness.

### 2.2. Resident Interview

As the subject of physical fitness, the relevant community residents and managers are selected to conduct questionnaire-style exchanges and face-to-face communication presented in this paper to fully understand the current urban residents' physical exercise methods, their understanding of the internal and external environment, and the needs of community sports facilities.

### 2.3. Questionnaire Survey and Statistics

The analysis and investigation of the awareness, demand, and satisfaction of urban residents are conducted on physical fitness, and the corresponding data are collected and summarized for statistics and analysis.

### 2.4. Telephone Survey

The telephone survey method was adopted to inquire the relevant contacts and telephone numbers of all the relevant information of the survey and conduct telephone surveys and information collection.

## 3. Simulation Experiment

For urban national physical fitness, its exercise methods under different conditions are different. The ant colony algorithm is introduced in this paper, taking inclement weather and haze weather as an example, fully analyzing the needs of urban national physical fitness, and conducting the corresponding simulation experiment [20].

### 3.1. Changes in the Fitness Concept of Urban Residents

With the in-depth implementation of related policies such as urban national fitness, especially the use of corresponding new media, such as Weibo and Douyin, people have a deep understanding and cognition of the science and necessity of physical exercise, especially for aerobic exercises, yoga exercises, etc., which are extremely important within a reasonable range of exercise and exercise intensity.

As far as the understanding of physical fitness is concerned, traditional walks and exercises are no longer popular, which are replaced by targeted aerobic exercises, large-scale square dancing, etc., which are demanding in venues and environments. At present, it is more common to be subhealthy under high work pressure, so the relevant environment needs to be considered to improve the safety and effectiveness of fitness.

Through related research and interviews, it can be seen that the distribution of physical fitness facilities can affect the fitness choices of urban residents, such as distance, openness of the venue, and diversification of content (whether there is a swimming pool, badminton hall, table tennis hall, basketball field, etc.), all of which have a certain impact.

### 3.2. Changes in the Understanding of Fitness Functions of Urban Residents

At present, the number of people in a subhealthy state is increasing. As the country and individuals demand more and more physical fitness, they are becoming more and more urgent. The fitness function of sports is considered to be the most effective and economical means to treat subhealth. It can exponentially save the consumption of medical resources and can be correlated with the individual's living habits and life events to form an individual's healthy life ecosystem. The fitness value of sports is not only embodied in promoting people's physical health but also effectively enhancing people's spiritual, psychological, and social health.

A survey on the understanding of the physical function of the fitness group of urban residents found that 83% of citizens believe that the function of sports is to keep fit, and 91% of the surveyors associate sports with people's mental health and believe that physical activity can regulate emotions, relieve pressure from life and work, and release bad emotions during exercise, especially for working people in a subhealthy state. At the same time, the functions of sports education and social promotion are gradually being valued.

### 3.3. Changes in the Choice of Fitness Venues for Urban Residents

In the context of the national urban ecological construction, the construction of the urban ecological environment has led to the greater development of ecological community resources. The current community construction, whether it is a mature community or a new community, puts the construction and improvement of the community's ecological environment as a priority, and at the same time, it is supplemented by the factors of community sports facilities and equipment. At present, the achievements of urban ecological sports environment construction have effectively expanded and revitalized community sports venues and facilities. (1) The construction of green space in the ecological community environment directly improves the living space of residents and at the same time enables residents to have a deeper understanding of community green space construction and functions and promotes its development in the direction of community ecological green space construction that integrates multiple activities and functions. The organic combination of community green space resources and community sports is an important direction of community ecological environment transformation in the future. (2) The construction of a community ecological environment incorporates sports venues with complete facilities, beautiful environments, and outstanding personalities. This measure guides mass sports out of traditional sports venues and toward urban ecological communities. The construction and improvement of the ecological environment have unconsciously guided and promoted the occurrence of this conscious exercise behavior of citizens. An open space, a group of fitness equipment, and a green fitness path can all realize diversified exercise behaviors.

The integration of the community ecological environment and community sports activities has enriched the physical fitness activities of community residents and added vitality to these outdoor fitness sports. Community residents broke through the traditional concept of fitness exercises in indoor stadiums, went more outdoors, toward nature, and started diversified sports activities. Traditional sports and fitness programs such as foot basket volleyball, badminton tennis, and swimming have certain requirements for venues and facilities, and more need to be carried out in indoor halls. With the improvement and perfection of the community ecological environment, the community ecological sports resources are recycled The system is gradually taking shape. More and more community residents like and enjoy outdoor aerobics fitness exercises. The fitness and sports activities that community residents are happy to participate in tend to be a green outdoor natural ecological environment that does not require special venues and facilities.

### 3.4. Analysis of Changes in Fitness Activities and Participation Methods of Urban Residents

According to the third survey on the status quo of mass sports, the sports event with the highest participation rate of residents ranked first is walking, followed by running, and third is the fitness path. The 6 sports activities residents hope most to participate in are walking, running, badminton, fitness path, square dancing, and swimming. According to this statistical result, activities such as walking, running, fitness trails, and badminton that require low levels of professionalism in exercise venues can be carried out independently in the green ecological environment of the community and have gradually developed into a higher frequency of exercise for community residents in sports activities.

Field observations and interviews learned that the design characteristics of fitness facilities and venues affect residents' choices of exercise behavior and methods. The fitness path is widely popular, mainly practicing running and walking; the small square, green space, and facilities are quiet and elegant, mainly for Tai Chi, diabolo, martial arts, skipping, and other exercise methods; large and medium-sized squares are magnificent and crowded, mainly developing squares in group activities such as dances and group dances; ecological sports resources are beautiful and pleasant, and the sports venues are relatively professional and attractive to people such as basketball, football, badminton, and table tennis.

The physicalization of the ecological community environment has made community residents' fitness participation methods more flexible and diversified, and indirectly has a great impact on community residents' personal exercise behaviors, family exercise behaviors, friend exercise behaviors, group exercise behaviors, and other sports participation methods. The impact stimulates the desire and enthusiasm of community residents to participate in sports and promotes the vigorous development of community residents' sports and fitness activities. The same survey results of the national fitness activities further illustrate that the development and construction of urban ecological sports resources invisibly cater to and meet the new needs of community residents' fitness methods, and it also has a certain value and significance for promoting national fitness.

### 3.5. Demand Analysis of Urban Residents' Fitness Activities

#### 3.5.1. Subjective and Objective Needs of Residents in Fitness Activities

First of all, the needs of urban residents and the corresponding physical fitness facilities provided by the city are evaluated and analyzed. For different and diversified needs, the investigation and analysis are mainly conducted subjectively and objectively.

As shown in the results in Figure 2, according to the results of the corresponding urban residents' physical fitness survey activities, the first is for “body building,” the second is to focus on “physical and mental health,” the third is to “relax the body and mind,” and the final is the selection related to “group activity” and “skill learning.”

For the fitness needs of urban residents, the relevant national, provincial, municipal, and local policies need to be integrated to form a complete set to meet the fitness needs of corresponding urban residents.

#### 3.5.2. The Residents' Cognitive and Behavioral Changes in Physical Exercise under Harsh (Smoggy) Environments and Analysis of Their Needs

1. Urban residents do not have enough knowledge or awareness about fitness under severe weather. More than 50% of urban residents believe that physical exercise is not possible under severe weather, and about 30% of residents believe that they can have choices, such as indoor activities. However, intense ball games are not allowed, which can be replaced with gentle exercises. Only a small number of people think that normal physical activities can be performed, as shown in Figure 3.
2. Under harsh conditions, on one hand, visibility is low, on the other hand, safety and health are not enough for sports, which is easy to cause too many physical health problems, especially for high-light physical fitness.
3. Under severe conditions, on one hand, visibility is low, and the air will be mixed with fine particles such as PM2.5. According to expert interviews, it is best not to engage in outdoor sports in this situation. Once the particular matter directly adheres to the respiratory tract and alveoli, it can cause rhinitis, bronchitis, and other diseases. If the air pollution is serious, it is even more likely to cause cancer than smoking. On the other hand, for sports, safety and health are not enough, and it is easy to cause too many physical health problems, especially for high and mild physical fitness.
4. Little change occurs to the frequency of residents' fitness activities due to inclement weather. From the survey of physical fitness habits of urban residents, it is found that more than 70% of residents have corresponding physical fitness habits themselves, mainly middle-aged and elderly people, but they generally choose corresponding external exercises. Only a small proportion of the people will insist on protecting themselves against inclement weather, and residents who do not participate in physical exercise or reduce the number of times account for about 20%, as shown in Figure 4.

Therefore, it can be seen that under severe conditions, urban residents' physical fitness has actually increased their demand for indoor venues. Meanwhile, it is worth noting that these physical exercises cannot be completed at home. The facilities need to be matched according to the corresponding need, and a suitable venue is selected for comprehensive physical exercise.

### 3.6. Analysis of the Supply of Urban Residents' Sports Activities

#### 3.6.1. Statistics of Facility Supply Resources for Residents' Sports Activities

Taking a certain city as an example, the corresponding physical exercise places in the city are calculated, as shown in Figure 5. These stadiums provide diversified exercise methods, meanwhile, the facilities of the stadiums are also satisfactory, with the convenient traffic. But in the meanwhile, the corresponding fees are higher.

The ant colony algorithm is used for calculations; based on the results of the calculations, we can see that there are more than 175 ways to provide sports, including table tennis, basketball, dance, aerobics, and yoga. In this way, there are both indoor and outdoor activities, and most places are generally free (Figure 6).

#### 3.6.2. Survey on the Service Supply of Residents' Sports Activities

Physical fitness activities of urban residents are spontaneous. With the gradual rise of various policies in recent years, various physical fitness venues have been continuously enriched, and the community and the government have gradually encouraged physical fitness.

### 3.7. Analysis of the Current Supply Structure's Satisfaction with Residents' Fitness Needs in Harsh Environments

#### 3.7.1. The Supply of Stadiums and Facilities which Cannot Meet the Needs of Residents for Fitness Activities

Through a comprehensive investigation, the current sports facilities and community-organized sports activities, and corresponding physical fitness services can hardly fully meet the physical fitness needs of the corresponding urban residents.

#### 3.7.2. Difficulty in Achieving Simultaneous Supply of the Space and Internal Air Quality of Existing Sports Facilities in Harsh Environments

For inclement weather, fully performing physical fitness exercises is hard in inclement weather, and more physical exercises need to be completed indoors. Therefore, this puts a higher demand on indoor fitness venues so as to meet the body-building needs of urban residents.

However, from the analysis of the supply of sports facilities, the proportion of indoor stadiums is not high. Commercially operated stadiums account for more than 85% of indoor stadiums, while the percentage of indoor stadiums in community cultural activity centers is lower. In the survey of whether indoor sports venues have air purification equipment, it is found that less than half of the venues that are equipped with air purification equipment are perceived by the survey subjects, and the proportion of air quality standards that can meet the air quality standards will be further reduced. This situation was also confirmed in the telephone survey (Figure 7). When asked “Can the fresh air system block PM2.5 particles?” and “How often should the dust filter of the filter system be replaced?” Most stadiums and gymnasiums have no clear inspection and maintenance records.

It can be seen from Figure 7 that it is difficult to meet the supply of sports facilities for urban residents. It is necessary to rely on the government to carry out reasonable resource allocation and activity organization of fitness facilities to form corresponding activity organizations. Through the calculation and analysis of the ant colony algorithm, urban residents have insufficient knowledge and awareness of physical fitness under severe weather. Physical fitness is more influenced by personal habits. The choice of venues for urban residents determines the way of physical fitness, chiefly including the following aspects: in harsh environments, urban residents generally do not easily change their physical fitness methods; for urban residents, it is hardly ensured that they carry out the indoor exercise consistent with outdoor exercises, which will change according to the environment; in the harsh environment, the supply-demand relationship between related fitness facilities and venues is still strained and cannot be satisfied. The simulation experiment proves that the ant colony algorithm is effective.

## 4. Conclusions

With the continuous development of the social economy, physical fitness has become an issue that has received more and more attention from urban residents. In response to these needs and problems, the ant colony algorithm is introduced by trial to analyze the sports facilities from the relationship between supply and demand by combing the concepts of urban residents' physical fitness; especially under severe conditions, urban residents have changed their need of physical fitness in a subjective and objective manner; thereby, the corresponding analysis results can be drawn to further improve the safety, health, and effectiveness of physical fitness. The results of simulation experiments show that the ant colony algorithm is effective and can support the prediction and analysis of the city's national sports and fitness demand.

## Figures and Tables

**Figure 1:** Schematic diagram of research ideas on the demand and supply of urban residents' fitness activities in harsh environments.

**Figure 2:** Schematic diagram of the subjective needs of Shanghai residents for fitness activities.

**Figure 3:** Schematic diagram of residents' perception of sports activities in inclement weather.

**Figure 4:** Survey on whether residents with fitness habits insist on participating in sports activities in inclement weather.

**Figure 5:** Distribution of community cultural activity centers.

**Figure 6:** Statistics of physical training place operated commercially.

**Figure 7:** Installation of the fresh air system and air purification equipment in stadiums.

## Data Availability

Data sharing is not applicable to this article as no datasets were generated or analysed during the current study.
